The article "Significance of the Expression of TC and TG Levels in the Initial Diagnosis and Treatment of SCLC Patients and Their Tie-In with Prognosis" was retracted in 2023. Reasons: signs of a paper mill; suspected computer-generated content; unreliable results or conclusions; concerns about the data.

# Significance of the Expression of TC and TG Levels in the Initial Diagnosis and Treatment of SCLC Patients and Their Tie-In with Prognosis

**DOI:** 10.1155/2022/1297072

**Published:** 2022-06-29

**Authors:** Qiankun Chen, Feng Tang, Haiping Zhang

**Affiliations:** ^1^Thoracic Surgery, Shanghai Pulmonary Hospital Affiliated to Tongji University, Shanghai 200082, China; ^2^Respiratory Medicine, Shanghai Pulmonary Hospital Affiliated to Tongji University, Shanghai 200082, China; ^3^Oncology, Shanghai Pulmonary Hospital Affiliated to Tongji University, Shanghai 200082, China

## Abstract

The article examines the expression of TC and TG levels in the initial diagnosis and treatment of SCLC patients and their tie-in with prognosis. Patients with SCLC are included in the case set, who are initially treated in the tumor center of our hospital from January 2020 to January 2021 and are confirmed by histopathology or cytology as the research subjects. 80 healthy volunteers are included in the control set, who received physical examination. All the enrolled patients received the first-line standard treatment plan, and the clinical data of all SCLC patients are inquired through the medical record file system of the hospital. At the initial diagnosis and treatment, the TG and TC levels of all patients and healthy persons are measured and recorded by blood biochemistry. For SCLC patients, the risk factors affecting the prognosis of patients with progression-free survival include newly diagnosed TC, TG levels, and tumor stage. Combined TC and TG detection can be used as indicators to predict the prognosis of the patients. TC and TG are significantly correlated with the prognosis of the patients with progression-free survival time. It is worthy of clinical application.

## 1. Introduction

Currently, lung carcinoma accounts for 30% of all carcinoma deaths in the world and is one of the most harmful carcinomas to human beings. Lung carcinoma is the carcinoma with the highest morbidity and mortality in China, posing a serious threat to the physical and mental health of the residents [1]. According to the pathological type, it can be divided into non-small-cell lung carcinoma and small-cell lung carcinoma (SCLC) [2]. SCLC is a neuroendocrine tumor derived from bronchial mucosal epithelial argentophilic cells. It contains relatively unique neurosecretory granules. After staining with neuron-specific enolase, it can be found to be significantly positive. Among all types of lung carcinoma, SCLC accounts for about 15%, and has the characteristics of high malignancy, short doubling time, extensive early metastasis, sensitivity to radiotherapy and chemotherapy, and easy recurrence and metastasis. At present, the clinical staging mainly refers to the method of the American Veterans Administration Lung carcinoma Association. According to the radiation field, it is divided into limited stage and light initiation. The median survival time of the limited stage SCLC patients is 18–24 months, and the 5-year survival rate is 10%–13%, patients with the extensive stage have a median survival of 9–10 months, and the 5-year survival rate is less than 5% [3]. Therefore, early diagnosis and early treatment are extremely important for SCLC patients. As one of the important components of lung tissues, lipids can be synthesized and broken down in the lungs. In the human body, blood lipids mainly play the role of energy supply, and their main role is to participate in the synthesis of cell membranes [4]. When lung carcinoma occurs, the proliferation of tumor cells is abnormally active, and the tumor cells continue to proliferate, and in this process, more energy and cell membrane synthesis are required. Therefore, the occurrence and development of lung carcinoma will be accompanied by abnormal lipid metabolism. However, the role and the pathways of lipid metabolism in the occurrence and development of lung carcinoma have not been fully studied, and the role of blood lipids in the prognosis of lung carcinoma is still unclear [5]. This paper collects the clinical data of patients with SCLC confirmed by histopathology or cytology in our hospital and studies the blood lipids of the SCLC patients. The tie-in between the level and the prognosis is to determine whether the blood lipid level during the initial treatment of small cell lung carcinoma affects the prognosis and to provide a theoretical basis for the clinical treatment of SCLC patients.

80 healthy volunteers who received physical examination in our hospital during the same period are selected and included in the control set, including 59 males and 21 females. The general clinical data such as age and gender are in contrast between the two sets, and there is no significant difference between the two sets. All patients signed informed consent, and this study is approved by the medical ethics committee of our hospital (ethics approval number: TJ IRB20201002).

Inclusion criteria include the following: (1) SCLC is diagnosed after bronchoscopy or a puncture histopathological examination; (2) the treatment regimens are carried out in accordance with the NC-CN guidelines [6]; and (3) there is no history of nausea and tumor. Exclusion criteria include the following: (1) pathologically diagnosed SCLC with squamous cell carcinoma or adenocarcinoma; (2) death due to non-lung carcinoma; (3) acute infection or dyslipidemia before treatment; (4) incomplete clinical data; and (5) participation in multiple researchers at the same time.

The remainder of this paper is organized as follows.  Section 2 presents the experimental method.  Section 3 provides the experimental result and Section 4 illustrates data analysis and result discussion. Finally, the conclusions of this study and some future recommendations are given in Section 5.

## 2. The Experimental Method

All the enrolled patients received the first-line standard treatment regimen for at least 4 courses. For the patients treated with the EP or EC regimen, one course of treatment lasted 21 days. And the patients are required to undergo a relevant imaging examination for two courses of treatment. The clinical data of all SCLC patients are queried through the hospital's medical record system, including the patient's name, age, gender, smoking status, BMI, TC and TG at the visit, treatment plan, surgery, time of diagnosis, and date of first progression.

During the initial diagnosis and treatment, 5 ml of cubital venous blood is collected from all participating researchers in the fasting state in the morning and centrifuged at 3 500 r/min for 10 min, and the centrifugation radius is 10 cm. The serum is collected for testing, and all patients' and health personnel's TG and TC levels are recorded.

In this article, all the data are organized, and all the databases are entered into SPSS 26.0 for data processing, and the measurement data is tested for normality. The multiset test is F, between sets is the *t-test*, and the nonnormality is the Mann–Whitney *U* test. The rate is expressed as %, and the test is the *χ2*. The tie-in between serum lipid TC and TG levels and prognosis in SCLC patients is examined by Pearson's correlation coefficient. The influencing factors are examined by multivariate logistic regression, the ROC curve is used to compare the diagnostic performance of TC and TG levels in the prognosis of SCLC, and the difference is considered statistically significant when *P* < 0.05.

## 3. The Experimental Results

### 3.1. Contrast of the Expression Levels of TC and TG between the Case Set and the Control Set

There are significant differences in the expression levels of TC and TG between the case set and the control set.  Table 1 shows the contrast of the expression levels of TC and TG between the case set and the control set.

### 3.2. Univariate Analysis of Clinical Data Differences in the Prognosis of SCLC Patients with Progression-Free Survival Time

Univariate results show that there are significant differences in the prognosis of SCLC patients with TC, TG, and tumor staging indicators in terms of the progression-free survival time. The progression survival time is significantly lower than that of TC < 5.5 mmol/L, TG < 1.7 mmol/L, and limited stage patients, and the difference is statistically significant (all *P* < 0.05). There is no significant difference between other clinical data (*P* > 0.05).  Table 2 shows the univariate analysis results of clinical data differences in the prognosis of SCLC patients with progression-free survival time.

### 3.3. Logistic Regression Multivariate Analysis of the Risk Factors Affecting the Prognosis of SCLC Patients with Progression-Free Survival Time

The multivariate analysis assignment takes the prognosis and progression-free survival time as the research dependent variable and combines the actual clinical situation to screen the model. TG > 1.7 mmol/L and the limited stage are risk factors affecting the prognosis of SCLC patients with progression-free survival time (*P* < 0.05).  Table 3 presents logistic regression multivariate analysis of the risk factors for progression-free survival time in patients with SCLC.

### 3.4. The Diagnostic Value of TC Combined with TG on the Prognosis and Survival of SCLC Patients

The area under the ROC curve of TC and TG levels for the evaluation of the progression-free survival time in SCLC patients is both>0.75, with high specificity and sensitivity, and the combined prediction is significantly higher than that of TC and TG alone. The area under the ROC curve is 0.775 and 0.759. There is a statistical difference between the three detection methods in the analysis and prediction model (*Z* = 2.235, *P* < 0.05).  Table 4 shows the diagnostic values of TC combined with TG on the prognosis of SCLC patients with progression-free survival time.  Figure 1 is the ROC curve of the diagnostic value of combined TG on the prognosis and survival of SCLC patients.

### 3.5. Analysis of the Tie-In between the Expression Levels of TC and TG in SCLC Patients and the Prognosis of Progression-Free Survival Time

There is a significant negative tie-in between the expression levels of TC and TG and the prognosis of progression-free survival in SCLC patients (*r* = -0.723,−0.829, both *P* < 0.05).  Table 5 shows the tie-in between TC and TG expression levels and the prognosis of progression-free survival in SCLC patients.  Figure 2 shows the tie-in between the TC expression level and prognosis of progression-free survival in SCLC patients.  Figure 3 presents the tie-in between the TG expression level and prognosis of progression-free survival in SCLC patients.

## 4. The Experimental Result Analysis

SCLC is a pathological type of lung carcinoma with a clinical incidence of about 15–20%. The occurrence of this disease is closely related to smoking and has high invasiveness after occurrence [7]. Due to its unique characteristics of neuroendocrine tumors, its clinical diagnosis is different from that of non-small cell lung carcinoma, such as paraneoplastic syndrome, abnormal secretion of antidiuretic hormone, and Lambert–Eaton myasthenic syndrome contrast with other pathological types of lung carcinoma. SCLC is more sensitive during chemotherapy and radiotherapy, but most SCLC have distant metastasis at the time of diagnosis, the prognosis is poor, and the 5-year survival rate is relatively low [8]. The main function of lipids in the human body is to provide energy for the operation of the body, and also to maintain cell integrity and many biological functions, such as cell growth and division in the body. Therefore, impaired lipid metabolism in the body may lead to the occurrence and development of some diseases. Neutral plasma fatty acids and lipids are collectively referred to as blood lipids [9]. Blood lipids are closely related to metabolic disorders of the lipid system in the body and cardiovascular diseases. It is clinically used as an indicator to monitor the process of metabolic health. A large number of epidemiological and experimental studies have found that factors affecting blood lipid levels include smoking, diet, and obesity, and may be closely related to the risk of carcinoma. In clinical practice, TC and TG are the main indicators for monitoring blood lipid levels.

With the gradual deepening of the research on the relationship between blood lipids and tumorigenesis, the detection of TC and TG is convenient and easy to obtain as a direct representative of human blood lipids. The results show that the expression levels of TC and TG in the case set are significantly higher than those in the control set (*P* < 0.05). This article finds that the results of the logistic regression model analysis show that TC > 5.5 mmol/L, TG > 1.7 mmol/L, and the limited stage are risk factors affecting the prognosis of SCLC patients (*P* *<* 0.05). In cells, the main function of cholesterol is to participate in and play an important role in the formation of the lipid valve domain, which contains a special membrane structure that constitutes the transport of normal cells and carcinoma cells. It is an organization center and is involved in a variety of pathophysiological processes, including cell apoptosis and signal transduction. Second, TC and TG are involved in interfering with fatty acid metabolism, thereby affecting tumor progression. The synthesis and decomposition of lipid fatty acids maintain energy balance and lipid accumulation in the body. Gabor pointed out the enzymes involved in fatty acid synthesis. It is highly expressed in carcinoma patients. In addition, in carcinoma cells, lipid valves can act on various classification signals and are related to many carcinoma-related molecules and adhesion molecules, and in the tumor microenvironment, lipid valves can be passed through autocrine or secreted growth factor receptors, by promoting cell growth and reproduction. Therefore, it is speculated that the expression of TC and TG blood lipids in the body can determine the reproduction of tumor molecules in the body. Therefore, this article uses TC and TG to evaluate the prognosis and survival of SCLC patients. The results show that the area under the ROC curve is > 0.75, with high specificity. The combined prediction is significantly higher than the area under the ROC curve of TC and TG detection by 0.775 and 0.759. There is a significant negative tie-in between the expression levels of TC and TG and the prognosis of progression-free survival time (*P*<0.05), suggesting that the combination of TC and TG can be used as a predictor of progression-free survival in SCLC patients. The main reason for the analysis is that excessive fat is the cause of the failure of the immune surveillance system composed of natural killer cells, like important immune cells in the body, which can resist and kill tumor cells, so high levels of TC TG can lead to an increased risk of metastasis in small-cell lung carcinoma through immune surveillance functions, thereby affecting the prognosis of patients.

## 5. Conclusion

To sum up, the levels of TC and TG at the initial diagnosis of SCLC patients are risk factors affecting the prognosis of patients with progression-free survival, and the combined detection of TC and TG can be used as indicators to predict the prognosis of patients. There is a significant tie-in with time, and it is worthy of clinical application.

Although this study has achieved certain results, it still has certain limitations. Because current studies have pointed out that there is a certain relationship between blood lipids and carcinoma, this study only selected TG and TC in blood lipids and did not examine all blood lipid indicators. The prediction of disease has a certain bias, so in future studies, the relationship between the prognosis of SCLC patients and blood lipids can be examined by expanding the sample size and indicators.

## Figures and Tables

**Figure 1:** ROC curve of the diagnostic value of combined TG on the prognosis and survival of SCLC patients.

**Figure 2:** Tie-in between the TC expression level and prognosis of progression-free survival in SCLC patients.

**Figure 3:** Tie-in between the TG expression level and prognosis of progression-free survival in SCLC patients.

**Table 1:** Contrast of the expression levels of TC and TG between the case set and the control set.

Set	Number of cases	TC	TG
Control set	80	4.32 ± 0.81	0.96 ± 0.31
Case set	90	5.91 ± 1.31	1.95 ± 0.53
*T*		−9.377	−14.628
*P*		<0.001	<0.001

**Table 2:** Univariate analysis of clinical data differences in the prognosis of SCLC patients with progression-free survival time.

Index		PFS (months)	*t*	*P*
Gender	Male (*n* = 62)	9.85 ± 1.23	−0.957	0.341
	Female (*n* = 28)	10.12 ± 1.26		
Age	>65 years old (*n* = 31)	9.89 ± 1.32	−0.236	0.814
	≤65 years old (*n* = 59)	9.96 ± 1.35		
Tumor stage	Limited period (*n* = 51)	12.59 ± 1.63	16.607	<0.001
	Extensive period (*n* = 39)	7.33 ± 1.28		
Distant metastasis	Yes (*n* = 21)	10.59 ± 1.57	−1.654	0.102
	No (*n* = 69)	11.19 ± 1.42		
Lymph node metastasis	Yes (*n* = 25)	8.99 ± 1.26	−1.847	0.068
	No (*n* = 65)	9.56 ± 1.33		
BIM classification	<18.5 kg/m^2^ (*n* = 20)	6.73 ± 1.02	−1.632	0.106
	18.5∼24.9 kg/m^2^ (*n* = 33)	10.69 ± 1.42		
	>24.9 kg/m^2^ (*n* = 37)	8.23 ± 1.34		
Smoking status	Yes (*n* = 62)	9.55 ± 1.36	−1.157	0.250
	No (*n* = 28)	9.91 ± 1.38		
HDL-C	<1.0 mmol/l (*n* = 42)	9.89 ± 1.42	1.286	0.202
	≥1.0 mmol/l (*n* = 48)	9.51 ± 1.38		
TC	>5.5 mmol/L (*n* = 47)	7.52 ± 1.15	−16.545	<0.001
	≤5.5 mmol/l (*n* = 43)	12.33 ± 1.59		
TG	>1.7 mmol/L (*n* = 39)	12.95 ± 1.69	23.209	<0.001
	≤1.7 mmol/l (*n* = 51)	6.13 ± 1.09		
Operation	Yes (*n* = 62)	10.15 ± 1.48	1.441	0.153
	No (*n* = 28)	9.68 ± 1.32		
Radiotherapy	Yes (*n* = 65)	10.25 ± 1.52	1.939	0.056
	No (*n* = 25)	9.56 ± 1.49		

**Table 3:** Logistic regression multivariate analysis of risk factors for progression-free survival time in patients with SCLC.

Index	Results of multivariate analysis					
	*β*	SE	Wald	OR	95% CI	*P*
TC	0.826	0.325	6.613	0.482	0.316∼0.532	0.003
TG	0.300	0.046	40.215	0.351	0.251∼0.513	0.005
Tumor stage	0.524	0.252	11.136	0.512	0.312∼0.755	0.001

**Table 4:** The diagnostic value of TC combined with TG on the prognosis of SCLC patients with progression-free survival time.

Index	Accuracy	Sensitivity	Specificity	AUC	Youden index
TC	81.00	80.00	76.60	0759 (0.594∼0.779)	0.560
TG	86.00	87.50	80.26	0.775 (0.662∼0.857)	0.681
Joint detection	97.00	97.50	94.20	0.957 (0.913∼0.969)	0.917

**Table 5:** Tie-in between TC and TG expression levels and the prognosis of progression-free survival in SCLC patients.

Index	Progression-free survival time	
	*r*	*P*
TC	0.562	<0.001
TG	0.857	<0.001

## Data Availability

The simulation experiment data used to support the findings of this study are available from the corresponding author upon request.
